# lncRNA ZEB1-AS1 inhibits high glucose-induced EMT and fibrogenesis by regulating the miR-216a-5p/BMP7 axis in diabetic nephropathy

**DOI:** 10.1590/1414-431X20209288

**Published:** 2020-04-09

**Authors:** Qingqing Meng, Xiaolin Zhai, Yi Yuan, Qing Ji, Pengyuan Zhang

**Affiliations:** Department of Nephrology, Luoyang Central Hospital Affiliated to Zhengzhou University, Luoyang, Henan, China

**Keywords:** ZEB1-AS1, miR-216a-5p, BMP7, Diabetic nephropathy, EMT, Fibrogenesis

## Abstract

Diabetic nephropathy (DN) is one of the leading causes of mortality in diabetic patients. Long non-coding RNA zinc finger E-box binding homeobox 1 antisense 1 (ZEB1-AS1) plays a crucial role in the development of various diseases, including DN. However, the molecular mechanism of ZEB1-AS1 in DN pathogenesis remains elusive. An *in vitro* DN model was established by treating HK-2 cells with high glucose (HG). Quantitative polymerase chain reaction (qRT-PCR) was utilized to detect the expression levels of ZEB1-AS1, microRNA-216a-5p (miR-216a-5p), and bone morphogenetic protein 7 (BMP7). Western blot assay was used to evaluate the protein levels of BMP7, epithelial-to-mesenchymal transition (EMT)-related proteins, and fibrosis markers. Additionally, the interaction among ZEB1-AS1, miR-216a-5p, and BMP7 was predicted by MiRcode (http://www.mircode.org) and starBase 2.0 (omics_06102, omicX), and confirmed by luciferase reporter assay. ZEB1-AS1 and BMP7 were down-regulated, while miR-216a-5p was highly expressed in kidney tissues of DN patients. Consistently, HG treatment decreased the levels of ZEB1-AS1 and BMP7, whereas HG increased miR-216a-5p expression in HK-2 cells in a time-dependent manner. ZEB1-AS1 upregulation inhibited HG-induced EMT and fibrogenesis. Furthermore, ZEB1-AS1 directly targeted miR-216a-5p, and overexpression of miR-216a-5p restored the inhibitory effects of ZEB1-AS1 overexpression on EMT and fibrogenesis. BMP7 was negatively targeted by miR-216a-5p. In addition, ZEB1-AS1 suppressed HG-induced EMT and fibrogenesis by regulating miR-216a-5p and BMP-7. lncRNA ZEB1-AS1 inhibited high glucose-induced EMT and fibrogenesis via regulating miR-216a-5p/BMP7 axis in diabetic nephropathy, providing a potential target for DN therapy.

## Introduction

Diabetic nephropathy (DN) is a common microvascular complication of diabetes and a major cause of end-stage renal disease (1). The typical characteristic of DN is the precipitation of extracellular matrix (ECM) in the mesangium and renal tubulo-interstitium along with thickening of glomerular and tubular basement membranes, eventually leading to glomerulosclerosis and tubulo-interstitial fibrosis (2). The increased ECM proteins including collagen, laminin, fibronectin, and proteoglycan, and ECM deposition lead to renal fibrosis (3). Although the main pathogenesis of DN has been identified, exploring effective molecular therapeutic targets is essential for DN treatment.

Epithelial-to-mesenchymal transition (EMT) is considered the main pathogenic factor of renal fibrosis, resulting in tubular atrophy as the main source of myofibroblasts (4,5). EMT presents as polarized epithelial cells that lose adhesion property and acquire mesenchymal phenotypes with invasive capacities (6). Accumulating evidence has demonstrated that the hallmark of EMT is the absence of epithelial-related protein (E-cadherin) and the increase of mesenchymal-related proteins (7). Renal fibrosis is the ultimate manifestation of DN, finally leading to end-stage renal disease (8). Increased ECM deposition leads to renal fibrosis. It has been reported that noncoding RNAs (ncRNAs) are new participants in the induction and regulation of EMT and kidney fibrosis (9,10). Therefore, it is meaningful to explore the roles of ncRNAs in the molecular mechanisms of EMT and fibrosis.

Long noncoding RNAs (lncRNAs) are noncoding transcripts with a length of more than 200 nucleotides (11). Increasing reports have indicated that lncRNAs modulate diverse biological processes, such as migration and invasion (12). Recently, studies reported that many lncRNAs played crucial roles in DN progression through direct pathogenesis or as indirect mediators of renal disease pathways (13). lncRNA zinc finger E-box binding homeobox 1 antisense 1 (ZEB1-AS1) is considered an oncogene in diverse tumors (14). ZEB1-AS1 facilitated cell migration and metastasis via targeting heterogeneous nuclear ribonucleoprotein D0 (AUF1) to activate ZEB1 expression in bladder cancer (15). Another study hinted that ZEB1-AS1 played an anti-fibrotic role in diabetic nephropathy (16). Nevertheless, the mechanism of ZEB1-AS1 in EMT and renal fibrosis of diabetic nephropathy remains unclear.

MicroRNAs (miRNAs) are highly conserved noncoding transcripts composed of 18–25 nucleotides (17). lncRNAs act as competitive endogenous RNAs (ceRNAs) that competitively bind to miRNAs (18). Recent studies indicated that miRNAs are involved in DN pathogenesis, including microRNA-216a (miR-216a) (19,20). However, the relationship between ZEB1-AS1 and miR-216a-5p in DN development is unknown.

Bone morphogenetic protein 7 (BMP7) has been reported to play a crucial role in renal disease and is absent in fibrogenic nephropathy (21). A number of studies have reported that BMP7 has a renoprotective effect in acute and chronic kidney disease models (22,23). Previous studies indicated that BMP7 could reduce diabetic renal injury, including podocyte dropout (24). Nevertheless, the role of BMP7 in DN requires further study.

In this study, we constructed a DN model in HK-2 cells. The role of ZEB1-AS1 on high glucose-triggered EMT and fibrosis was studied. We further explored the underlying mechanisms of ZEB1-AS1 in DN pathogenesis.

## Materials and Methods

### Tissue samples

Kidney tissues were collected from kidney biopsies from DN patients (n=20) and age-matched healthy volunteers (n=20) from Luoyang Central Hospital Affiliated to Zhengzhou University. The research was authorized by the Ethics Committee of Luoyang Central Hospital Affiliated to Zhengzhou University. All participatants signed a written informed consent.

### Cell culture

HK-2 cells were obtained from American Type Culture Collection (ATCC, USA). Cells were incubated with Dulbecco's Modified Eagle Medium (DMEM; Sigma-Aldrich, USA) supplemented with 10% fetal bovine serum (FBS; Gibco, USA) at 37°C with 5% CO_2_. Then, HK-2 cells were treated with normal glucose (NG, 5.5 mM glucose supplemented with 24.5 mM mannitol) or high glucose (HG, 30 mM glucose) for 12, 24, and 48 h.

### Cell transfection

Cell transfection was carried out by Lipofectamine 2000 (Invitrogen, USA). Specific vectors and oligonucleotides were as follows: ZEB1-AS1 overexpression vector (ZEB1-AS1), overexpression empty vector (pcDNA), miR-216a-5p mimic (miR-216a-5p), mimic negative control (miR-NC), small interfering RNA (siRNA) against BMP7 (si-BMP7), and siRNA negative control (si-NC). All sequences were synthesized by RiboBio (China).

### Quantitative polymerase chain reaction (qRT-PCR)

Total RNA was extracted from kidney tissues and HK-2 cells using Trizol reagent (Life Technologies Corp., USA). Then, cDNA was generated using High-Capacity cDNA Reverse Transcription Kits (Bio-Rad, USA) or miScript Reverse Transcription Kit (Qiagen, Germany). Finally, the expression levels of mRNA were monitored by SYBR Premix Ex Taq II (Takara, China). Glyceraldehyde-3-phosphate dehydrogenase (GAPDH) and U6 were used as standardized references. Primers were as follows: ZEB1-AS1-Forward: 5′-CCGTGGGCACTGCTGAAT-3′, ZEB1-AS1-Reverse: 5′-CTGCTGGCAAGCGGAACT-3′; miR-216a-5p-Forward: 5′-ACATCCTCGGCCAGTAAGACTG-3′, miR-216a-5p-Reverse: 5′-GTCGACCAGATTGCGTTCG-3′; BMP7-Forward: 5′-TCGGCACCCATGTTCATGC-3′, BMP7-Reverse: 5′-GAGGAAATGGCTATCTTGCAGG-3′; GAPDH-Forward: 5′-AGCCACATCGCTCAGACA-3′, GAPDH-Reverse: 5′-GCCCAATACGACCAAATCC-3′; 18S rRNA-Forward: 5′-AAACGGCTACCACATCCA-3′, 18S rRNA-Reverse: 5′-CACCAGACTTGCCCCTCCA-3′; U6-Forward: 5′-CTCGCTTCGGCAGCACA-3′, U6-Reverse: 5′-AACGCTTCACGAATTTGCGT-3′.

### Western blot assay

After extracting the proteins in cells using RIPA buffer (Invitrogen), the protein concentration was detected. After separating the protein samples by sodium dodecyl sulfate polyacrylamide gel electrophoresis (SDS-PAGE), the proteins were transferred to polyvinylidene fluoride membranes (Millipore, USA). Subsequently, after soaking for 2 h in 5% skim milk, the membranes were incubated with primary antibodies overnight at 4°C. Then, the membranes were coated with rabbit secondary antibody (1:4,000; Abcam, UK) for 2 h at 37°C. The protein bands were observed using enhanced chemiluminescence reagents (Millipore). The primary antibodies included E-cadherin (1:1,000; Abcam), vimentin (1:1,000; Abcam), α-smooth muscle actin (α-SMA) (1:1,000; Abcam), fibronectin (FN) (1:1,000; Abcam), collagen I (Col I) (1:1,000; Abcam), collagen IV (Col IV) (1:1,000; Abcam), BMP7 (1:1,000; Abcam), and GAPDH (1:1,000; Abcam).

### RNA isolation of nuclear and cytoplasmic fractions

The subcellular localization of ZEB1-AS1 was assessed using the PARIS Kit (Invitrogen) according to the manufacturer's protocol. U6 and 18S rRNA were used as positive control for nuclear and cytoplasmic fractions, respectively.

### Luciferase reporter assay

The fragment of ZEB1-AS1 (WT-ZEB1-AS1) or BMP7 3′ UTR (BMP7-3′UTR-WT) containing the predicted binding sites of miR-216a-5p and the mutant fragment (MUT-ZEB1-AS1 or BMP7-3′UTR-MUT) were inserted into pGL3 plasmids (Promega, USA). Subsequently, the recombinant vectors and miR-216a-5p or miR-NC were cotransfected into HK-2 cells with Lipofectamine 2000 (Invitrogen). Luciferase activity was analyzed using the Dual-Luciferase Reporter Assay System (Promega).

### Statistical analysis

Data are reported as means±SD from three independent experiments. Statistical significance was calculated by Student's *t*-test or one-way analysis of variance. Statistical analysis was carried out using Graphpad Prism 7.0 software (GraphPad, USA). Differences were considered to be statistically significant at P<0.05.

## Results

### ZEB1-AS1 was down-regulated and miR-216a-5p was upregulated in DN kidney tissues and HG-induced HK-2 cells

Firstly, we examined the expression levels of ZEB1-AS1 and miR-216a-5p in kidney tissues using qRT-PCR. The results showed that ZEB1-AS1 expression was significantly lower, while miR-216a-5p expression was significantly higher in kidney tissues of DN patients than in healthy controls (Figure 1A and B). In addition, we established a DN model *in vitro* by incubating HK-2 cells in 30 mM glucose. The results of qRT-PCR showed that HG treatment significantly decreased the expression of ZEB1-AS1 and increased the expression of miR-216a-5p in a time-dependent manner (Figure 1C and D). These data indicated that ZEB1-AS1 and miR-216a-5p might play roles in the progression of DN.

**Figure 1:** Expression levels of ZEB1-AS1 and miR-216a-5p in diabetic nephropathy (DN) kidney tissues and high glucose (HG)-induced HK-2 cells. **A** and **B**, Expression levels of ZEB1-AS1 and miR-216a-5p were examined in kidney tissues of DN patients and healthy volunteers by qRT-PCR. **C** and **D**, Expression levels of ZEB1-AS1 and miR-216a-5p were measured in HK-2 cells incubated with normal glucose (NG) or HG for 12, 24, or 48 h, respectively. Data are reported as means±SD. *P<0.05 (ANOVA).

### Overexpression of ZEB1-AS1 inhibited HG-induced EMT and fibrogenesis in HK-2 cells

To explore the functional role of ZEB1-AS1 in DN progression, HK-2 cells were transfected with pcDNA or ZEB1-AS1 and then stimulated with normal glucose (5.5 mM) or high glucose (30 mM) for 48 h. QRT-PCR revealed that ZEB1-AS1 expression was significantly increased in the ZEB1-AS1 group compared with the pcDNA group (Figure 2A). The results of western blot analysis showed that the protein level of EMT-related epithelial marker (E-cadherin) was reduced and the protein levels of EMT-related mesenchymal markers (α-SMA and vimentin) were increased in the HG group compared with the NG group, while ZEB1-AS1 overexpression impeded HG-induced EMT (Figure 2B). Furthermore, HG treatment significantly increased the protein levels of fibrosis markers (FN, Col I, and Col IV), whereas ZEB1-AS1 overexpression reduced the expression of fibrosis-related proteins (Figure 2C). Taken together, these data indicated that overexpression of ZEB1-AS1 inhibited HG-induced EMT and fibrogenesis in HK-2 cells.

**Figure 2:** Overexpression of ZEB1-AS1 inhibited high glucose (HG)-induced epithelial-to-mesenchymal transition (EMT) and fibrogenesis in HK-2 cells. **A**, Expression level of ZEB1-AS1 was detected in HK-2 cells transfected with pcDNA or ZEB1-AS1. **B**, Western blot assay was carried out to measure the protein levels of EMT-related markers (E-cadherin, α-SMA, and vimentin) in HK-2 cells transfected with pcDNA or ZEB1-AS1 and then treated with normal glucose (NG) or HG for 48 h. **C**, Western blot assay was performed to test the protein levels of fibrosis markers (FN, Col I, and Col IV) in HK-2 cells transfected with pcDNA or ZEB1-AS1 and then treated with NG or HG for 48 h. Data are reported as means±SD. *P<0.05 (ANOVA).

### ZEB1-AS1 regulated HG-induced EMT and fibrogenesis by directly targeting miR-216a-5p in HK-2 cells

In order to determine the subcellular localization of ZEB1-AS1 in HK-2 cells, we performed nuclear and cytoplasmic fraction assays. The results showed that ZEB1-AS1 was principally distributed in the cytoplasm of HK-2 cells (Figure 3A). miRcode online database was used to predict the putative targets of ZEB1-AS1, and miR-216a-5p was selected as the research object (Figure 3B). Subsequently, luciferase reporter assay was carried out to verify whether miR-216a-5p was a target of ZEB1-AS1. The results revealed that mature miR-216a-5p remarkably inhibited the luciferase activity of WT-ZEB1-AS1 reporter, but did not restrain the luciferase activity of MUT-ZEB1-AS1 reporter (Figure 3C). Meanwhile, the expression of miR-216a-5p was significantly enhanced in HK-2 cells treated with HG compared to the NG group and upregulation of ZEB1-AS1 significantly suppressed miR-216a-5p expression compared to the HG+pcDNA group (Figure 3D). In addition, the protein levels of EMT and fibrosis-related markers were examined by western blot assay in HG-treated HK-2 cells transfected with pcDNA, ZEB1-AS1, ZEB1-AS1+miR-NC, or ZEB1-AS1+miR-216a-5p, respectively. The results showed that overexpression of ZEB1-AS1 induced a significant increase of E-cadherin protein level and a decrease of protein levels of α-SMA and vimentin in HG-stimulated HK-2 cells, whereas the changes of EMT-related proteins were recovered after upregulation of miR-216a-5p (Figure 3E). Consistently, upregulation of ZEB1-AS1 markedly suppressed the expression of fibrosis-related proteins (FN, Col I, and Col IV), while the effects were abolished by upregulating miR-216a-5p (Figure 3F). All these data indicated that ZEB1-AS1 directly targeted miR-216a-5p and overexpression of miR-216a-5p restored the inhibitory effects of ZEB1-AS1 overexpression on EMT and fibrogenesis in HK-2 cells.

**Figure 3:** ZEB1-AS1 directly targeted miR-216a-5p in HK-2 cells. **A**, Expression of ZEB1-AS1 in the nuclear and cytoplasmic fractions was detected by qRT-PCR. **B**, The putative binding sites between ZEB1-AS1 and miR-216a-5p are exhibited. **C**, Luciferase reporter assay was used to analyze the luciferase activity in HK-2 cells cotransfected with wild type WT-ZEB1-AS1 or mutant MUT-ZEB1-AS1 and miR-216a-5p mimic or miR-NC (negative control). **D**, QRT-PCR was applied to examine the expression of miR-216a-5p in HK-2 cells treated with normal glucose (NG) or high glucose (HG) and HG-treated HK-2 cells transfected with pcDNA or ZEB1-AS1. **E** and **F**, HG-induced HK-2 cells were transfected with pcDNA, ZEB1-AS1, ZEB1-AS1+miR-NC, or ZEB1-AS1+miR-216a-5p. The protein levels of EMT-related markers (E-cadherin, α-SMA, and vimentin) and fibrosis markers (FN, Col I, and Col IV) were detected by western blot analysis. Data are reported as means±SD. *P<0.05 (*t*-test or ANOVA).

### BMP7 was a target of miR-216a-5p in HK-2 cells

Bioinformatics software StarBase 2.0 was applied to predict the potential targets of miR-216a-5p, and BMP7 was selected as a putative target (Figure 4A). Luciferase reporter assay demonstrated that mature miR-216a-5p reduced the luciferase activity of BMP7-3′UTR-WT reporter, but did not affect the luciferase activity of BMP7-3′UTR-MUT reporter (Figure 4B). Additionally, BMP7 expression was measured in kidney tissues. The result of qRT-PCR showed that BMP7 expression was down-regulated in kidney tissues of DN patients compared with healthy controls (Figure 4C). The results of qRT-PCR and western blot assay exhibited that high glucose significantly suppressed mRNA and protein levels of BMP7 in a time-dependent manner (Figure 4D and E). Furthermore, mRNA and protein levels of BMP7 were detected in HK-2 cells transfected with miR-NC or miR-216a-5p, respectively. These results suggested that the mRNA and protein levels of BMP7 were significantly decreased in HK-2 cells transfected with miR-216a-5p mimic compared with the miR-NC group (Figure 4F and G). These data demonstrated that BMP7 was a target of miR-216a-5p and was negatively regulated by miR-216a-5p in HK-2 cells.

**Figure 4:** BMP7 was a target of miR-216a-5p in HK-2 cells. **A**, Predicted binding sites of miR-216a-5p and BMP7 are shown. **B**, HK-2 cells were cotransfected with BMP7-3′UTR-WT or BMP7-3′UTR-MUT and miR-216a-5p mimic or miR-NC, then luciferase activity was evaluated by the luciferase reporter assay. **C**, Expression of BMP7 was measured in normal kidney tissues and kidney tissues with diabetic nephropathy (DN) by qRT-PCR. **D** and **E**, mRNA and protein levels of BMP7 were detected in HK-2 cells treated with normal glucose or high glucose for 12, 24 or 48 h, respectively. **F** and **G**, mRNA and protein levels of BMP7 were examined in HK-2 cells transfected with miR-NC or miR-216a-5p, respectively. Data are reported as means±SD. *P<0.05 (t-test or ANOVA).

### ZEB1-AS1 suppressed HG-induced EMT and fibrogenesis by targeting BMP7

To investigate the relationship among ZEB1-AS1, miR-216a-5p, and BMP7, HK-2 cells were transfected with pcDNA, ZEB1-AS1, ZEB1-AS1+miR-NC, or ZEB1-AS1+miR-216a-5p. The results showed that upregulation of ZEB1-AS1 drastically increased the mRNA and protein levels of BMP7, while the changes of BMP7 expression were recuperated after transfection with miR-216a-5p (Figure 5A and B). In addition, HG-treated HK-2 cells were transfected with pcDNA, ZEB1-AS1, ZEB1-AS1+si-NC, or ZEB1-AS1+si-BMP7, and the protein levels of EMT and fibrosis-related markers were measured using western blot assay. The results showed that overexpression of ZEB1-AS1 significantly inhibited HG-induced EMT, which was counteracted after transfection with si-BMP7 (Figure 5C). The expression levels of fibrosis-related proteins (FN, Col I, and Col IV) were significantly reduced in the HG+ZEB1-AS1 group compared to the HG+pcDNA group, which were restored by down-regulating BMP7 (Figure 5D). All these data indicated that ZEB1-AS1 regulated BMP7 expression by targeting miR-216a-5p and suppressed HG-induced EMT and fibrogenesis by targeting BMP7 in HK-2 cells.

**Figure 5:** ZEB1-AS1 suppressed high glucose (HG)-induced epithelial-to-mesenchymal transition (EMT) and fibrogenesis by upregulating BMP7. **A** and **B**, HK-2 cells were transfected with pcDNA, ZEB1-AS1, ZEB1-AS1+miR-NC (negative control), or ZEB1-AS1+miR-216a-5p, and the mRNA and protein levels of BMP7 were estimated using qRT-PCR and western blot assay, respectively. **C** and **D**, HG-stimulated HK-2 cells were transfected with pcDNA, ZEB1-AS1, ZEB1-AS1+si-NC, or ZEB1-AS1+si-BMP7, and the protein levels of EMT-related markers (E-cadherin, α-SMA, and vimentin) and fibrosis markers (FN, Col I, and Col IV) were measured by western blot analysis. Data are reported as means±SD. *P<0.05 (ANOVA).

## Discussion

Despite advances in treatment and research, the prognosis of DN is still very poor. Research has shown that EMT is the core of the underlying pathology of tubulointerstitial fibrosis in diabetic nephropathy (25). However, the molecular mechanisms of DN have not been fully studied. Increasing evidence has shown that ZEB1-AS1 is an oncogene in diverse malignancies via increasing ZEB1 expression (26). ZEB1-AS1 expression was enhanced in pulmonary fibrosis and promoted TGF-β1-induced fibrogenesis through ZEB1-mediated EMT by sponging miR-141-3p (27). Conversely, ZEB1-AS1 knockdown increased HG-induced ECM accumulation through down-regulating ZEB1 expression, leading to renal fibrosis in DN (16). In our, HG treatment distinctly increased the protein levels of mesenchymal markers and fibrosis markers. ZEB1-AS1 was down-regulated in DN. In addition, overexpression of ZEB1-AS1 inhibited EMT and fibrogenesis triggered by HG in HK-2 cells.

Accumulating evidence indicates that lncRNAs competitively bind with miRNAs to regulate target genes expression (28). Online forecasting software predicted that miR-216a-5p might be a target of ZEB1-AS1. Moreover, a previous study suggested that TGF-β promotes miR-216a expression in renal mesangial cells (29). In this study, miR-216a-5p expression was elevated in DN tissues, which was in line with previous reports. Furthermore, ZEB1-AS1 directly targeted miR-216a-5p and modulated EMT and fibrogenesis via sponging miR-216a-5p.

BMPs are classified as a superfamily associated with TGF-β (30). Accumulation of ECM proteins induced by TGF-β are hallmarks of diabetic nephropathy (31). Feng et al. (32) found that the protein expression of BMP7 was down-regulated in HG-induced DN. BMP7 might ameliorate DN and renal fibrosis by upregulating the expression of Ski-related novel protein N (SnoN) (33). Lv et al.(34) demonstrated that mesenchymal stem cells attenuate glomerular fibrosis by suppressing TGF-β/Smad signaling pathway through increasing BMP7. In the present study, miR-216a-5p directly targeted BMP7 and negatively modulated BMP7 in HK-2 cells. ZEB1-AS1 regulated BMP7 expression by targeting miR-216a-5p, and suppressed HG-induced EMT and fibrogenesis by elevating BMP7 expression in HK-2 cells.

In conclusion, ZEB1-AS1 could regulate BMP7 expression by functioning as a sponge of miR-216a-5p. Additionally, ZEB1-AS1 ameliorated high glucose-induced EMT and fibrogenesis by mediating miR-216a-5p and BMP7. These results suggested that the ZEB1-AS1/miR-216a-5p/BMP7 axis might be a potential therapeutic target for DN.
